# The role community‐based healthcare providers play in managing hard‐to‐heal wounds

**DOI:** 10.1111/iwj.14402

**Published:** 2023-09-15

**Authors:** Dimitri Beeckman, Matthew Cooper, Emily Greenstein, Patricia Idensohn, Robert J. Klein, Norbert Kolbig, Kimberly LeBlanc, Catherine Milne, Terry Treadwell, Dot Weir, Wendy White

**Affiliations:** ^1^ Skin Integrity Research Group (SKINT), University Centre for Nursing and Midwifery, Department of Public Health and Primary Care Ghent University Ghent Belgium; ^2^ Swedish Centre for Skin and Wound Research (SCENTR), School of Health Sciences Örebro University Örebro Sweden; ^3^ 3M Health Care St. Paul Minnesota USA; ^4^ Sanford Health Fargo North Dakota USA; ^5^ CliniCare Medical Centre Ballito South Africa; ^6^ Department of Surgery University of South Carolina School of Medicine Greenville South Carolina USA; ^7^ University Hospital Düsseldorf Düsseldorf Germany; ^8^ KDS Professional Consulting Ottawa Ontario Canada; ^9^ Connecticut Clinical Nursing Associates, LLC Bristol Connecticut USA; ^10^ Wound Care Solutions Montgomery Alabama USA; ^11^ Saratoga Hospital Center for Wound Healing and Hyperbaric Medicine Saratoga Springs New York USA; ^12^ Wendy White WoundCare Murwillumbah New South Wales Australia

**Keywords:** chronic wound, community healthcare provider, hard‐to‐heal wound, wound dressing, wound healing

## Abstract

It is common for community‐based healthcare providers (CHPs)—many of whom have not received specialised training in wound care—to deliver initial and ongoing management for various wound types and diverse populations. Wounds in any setting can rapidly transition to a stalled, hard‐to‐heal wound (HTHW) that is not following a normal healing trajectory. Failure to recognise or address issues that cause delayed healing can lead to increased costs, healthcare utilisation and suffering. To encourage early intervention by CHPs, a panel of wound care experts developed actionable evidence‐based recommendations for CHPs delineating characteristics and appropriate care in identifying and treating HTHWs. A HTHW is a wound that fails to progress towards healing with standard therapy in an orderly and timely manner and should be referred to a qualified wound care provider (QWCP) for advanced assessment and diagnosis if not healed or reduced in size by 40%–50% within 4 weeks. HTHWs occur in patients with multiple comorbidities, and display increases in exudate, infection, devitalised tissue, maceration or pain, or no change in wound size. CHPs can play an important initial role by seeing the individual's HTHW risk, addressing local infection and providing an optimal wound environment. An easy‐to‐follow one‐page table was developed for the CHP to systematically identify, evaluate and treat HTHWs, incorporating a basic toolkit with items easily obtainable in common office/clinic practice settings. A flow chart using visual HTHW clinical cues is also presented to address CHPs with different learning styles. These tools encourage delivery of appropriate early interventions that can improve overall healthcare efficiency and cost.

## 1 INTRODUCTION

Many people with wounds initially seek care from their community‐based healthcare providers (CHPs) who are often not specialised in wound care.^1^, ^2^, ^3^, ^4^ Wounds are also initially treated by individuals themselves and their circles of care.^2^, ^5^ Despite the rapidly growing prevalence and burden of wounds, a relatively small segment of wounds is treated by a qualified wound care provider (QWCP).^3^ Types of providers caring for wounds are described in Figure 1.

**FIGURE 1:** People providing wound care.

Variable levels of care can cause individuals' wounds to rapidly become stalled, not following the normal or desired trajectory of healing, and develop into a hard‐to‐heal wound (HTHW).^6^ A HTHW is defined as any wound that has not healed by 40%–50% after 4 weeks of good standard of care (SOC).^7^ HTHWs translate into an increased financial burden to the healthcare system (staff time, dressings and dressing supply usage and related medications costs) and increased cost to the individual (lost time from work, dressing supply costs and medication costs), as well as a humanistic burden including pain, emotional and physical distress, anxiety, sleep disturbance, reduced mobility, social isolation, and even disabilities and amputation.^8^, ^9^, ^10^, ^11^, ^12^, ^13^

Although delayed healing is common, it is frequently not recognised early enough by the CHP or patient, posing a major problem that increases cost and healthcare utilisation.^14^ In addition, CHPs may lack appropriate dressing materials in their practice to provide good SOC wound treatment. Failure to adequately address wounds not progressing towards healing increases the subsequent risk of non‐healing and places the patient at increased risk of wound complications.^15^ For example, if oedema is not controlled, a small skin tear on a lower limb of a patient with chronic stasis can quickly become chronic and complex with the potential to be a HTHW.^16^

While simple wounds that result from an injury can in most cases be successfully treated by a CHP, patients with a HTHW should be referred early to a QWCP.^7^ QWCPs are medical professionals, including nurses, physicians, surgeons, podiatrists and physical therapists, who have received specialised wound care training and certification (differing by care setting and country) and who have access to advanced wound care treatments and technologies not typically available in a primary healthcare facility.

Many situations stall the referral process and prolong the time between initial wound presentation and a visit to a QWCP or multidisciplinary wound care team. In all cases, CHPs can play a critical initial role by providing a thorough assessment and good standard wound care to help prevent deterioration and assist in reversing the trajectory towards healing. The aim of this publication is to provide evidence‐based wound care recommendations and suggestions for toolkit items within a wound healing framework that can easily be adopted into a CHP's practice for timely prevention and treatment of HTHWs.

## 2 METHODS

An advisory panel of QWCP experts met to discuss and develop simplified recommendations for managing HTHWs. The sponsor of this panel, 3M Health Care, invited panel members based on their clinical experience in wound care. Panel members were selected from Europe, North America, Australia and Africa. The advisory panel meeting was held in Atlanta, GA, between 17 and 18 June 2022. The participants consisted of eight nurses, one physiotherapist and three physicians, all with extensive experience and specialisation in wound care. Three members of the panel attended remotely, and the remainder met in person. The meeting was chaired by a moderator (author DB) and recorded for follow‐up. During the meeting, each panellist discussed the relevant literature, presented their individual clinical experiences and made suggestions for improving management of HTHWs.

The information presented during the meeting was summarised by a medical writer into an outline that was distributed to panel members for input. Follow‐up communication with the panel members continued via e‐mail and remote online meetings to review and solicit input on each draft. In cases of ambiguity in editing, the moderator determined the final text to be included in the manuscript. The final draft of this manuscript was approved by all panel members.

## 3 RESULTS

Following is a description of HTHWs along with practical, evidence‐based SOC wound care recommendations developed by panel members for any CHP who provides wound care. Instituting these recommendations into practice could make giant strides towards HTHW prevention and positive treatment outcomes.

### 3.1 Healing versus non‐healing (hard‐to‐heal) wounds

Acute wounds normally heal within 4–6 weeks with appropriate care. An expected healing trajectory that can be applied by clinicians to all wounds is 40%–50% wound size reduction at 4 weeks.^7^ By contrast, HTHWs are wounds that have not shown approximately 40%–50% wound size reduction within 4 weeks of evidence‐based SOC.

Multiple intrinsic and exogenous factors can cause dysregulation of the normal stages of healing in all wound types leading to HTHWs (Table 1). Most HTHWs are determined as “healable”, meaning they have adequate blood supply and the cause(s) can be treated. However, a small fraction of HTHWs are “non‐healable” as they have an inadequate blood supply and/or a cause that cannot be corrected or treated. Other HTHWs are deemed “maintenance” if there is an adequate blood supply to heal the wound, but the patient cannot or will not follow the plan of care and/or the healthcare system does not have appropriate resources.^17^ The focus of this publication is on the prevention and management of HTHWs that are considered “healable”.

**TABLE 1:** Wound types that have the potential to become hard to heal.

Acute		Chronic		
Surgical wounds	Traumatic wounds	Diabetic foot ulcers	Venous insufficiency ulcers	Arterial leg ulcers
Burns	Skin tears	Pressure injuries	Moisture‐associated skin damage	Malignant wounds
Spider, snake and dog bites	Crush, stab, degloving and gunshot wounds	Atypical wounds	Mixed arterial/venous vascular ulcers	Fungating wounds

#### 3.1.1 Recommendations for optimal standard of care in preventing and managing HTHWs

Recommendation 1 Predict hard‐to‐heal status early, by identifying and addressing, when possible, person‐related factors known to delay wound healing.

In addition to wound characteristics that predict hard‐to‐heal status, early identification of the type of person with a higher risk of having a HTHW is critical in preventing deterioration of the wound. Usually, HTHWs occur on elderly patients and/or patients with comorbidities, including those listed in Figure 2. Patient and wound complexity increase the likelihood of hard‐to‐heal status.

Recommendation 2 Use clinical signs to identify a HTHW as early as possible.

**FIGURE 2:** Person‐related risk factors associated with HTHWs.^7^, ^12^, ^51^

Knowledge of the major clinical indicators of failing wound treatment is essential for early intervention. Biofilm, a microbial colony encased in a self‐produced polysaccharide matrix, is known to be present in most HTHWs.^18^, ^19^ Biofilms increase the risk of infection and are associated with the stalled healing of HTHWs due to the production of destructive enzymes and toxins that promote a chronic inflammatory state within the wound.^20^

Clinical signs of biofilm typically mirror clinical signs of HTHWs, which are listed in Table 2. Early recognition of these subtle clinical signs and prompt referral of patients to receive biofilm‐based wound management are vital for timely wound healing.

Recommendation 3 Refer patients to a QWCP as soon as a HTHW is suspected, that is, before or at 4 weeks if not healed or surface area not reduced by 40%–50%.

**TABLE 2:** Clinical indicators of HTHWs.^7^, ^14^, ^20^

Increase in devitalised tissue
Poor granulation tissue or hypergranulation tissue that bleeds easily
Progression or recurrent infection, not responsive to appropriate antimicrobial treatment
Increase in exudate/moisture
Increase in maceration
Delayed healing despite excellent SOC
Low‐level erythema
Overall wound deterioration
Increased or new onset pain

Abbreviation: SOC, standard of care.

Whenever a HTHW is suspected, the earliest possible referral to a QWCP or multidisciplinary wound care team is recommended if the wound fails to progress.^2^, ^15^ While the traditional timeline for classifying a HTHW has been 4–12 weeks, the current literature overwhelmingly supports quicker identification and intervention by 4 weeks.^7^, ^20^, ^21^, ^22^ A slow or non‐healing trajectory can be predicted before 4 weeks with a basic understanding of normal wound healing progression and factors that lead to impaired healing.^15^, ^23^, ^24^

Recommendation 4 Perform a thorough holistic patient, wound and periwound assessment, including basic bedside vascular screening examinations and tests if applicable.

Holistic patient assessment, wound assessment, accurate diagnosis, treating underlying causes, thorough wound bed preparation and ongoing evaluation of the outcomes of treatment interventions are cornerstones of effective SOC wound management.^25^, ^26^ Holistic patient assessment is a patient‐centred approach that identifies whole patient needs and past medical and surgical history, assesses the anatomy, and records the wound history.^25^ The wound assessment should include a detailed description of the wound and accurate measurements. Observations, actions, interactions, interventions and outcomes should be documented in detail, including dates, times and photographs. A structured wound assessment should also include a description of the periwound integrity, which can be an important determinant in decreasing wound size.^27^

Assessing blood supply to a wound is recommended in cases where vascular disease, either arterial or venous, is suspected.^28^ This includes palpating the dorsalis pedis, posterior tibial and/or peroneal nerve, as well as performing the capillary refill test and a pallor/rubor test (at a minimum) or an audible waveform (if a handheld Doppler is available). If any of these tests cannot be performed, or abnormalities are detected during tests, patients should be referred to a QWCP.

Pathologies underlying wounds differ vastly, and the foundation of successful treatment lies in ensuring, when possible, that this is corrected or addressed by use of pressure relief, offloading, revascularisation and/or compression.^29^ Arterial supply should be optimised to the extent possible.

Recommendation 5 Deliver best practice standard of care when treating any wound.

With the growing prevalence of wounds, CHPs play an increasingly important role in wound management. The fundamental principle in wound management across healthcare settings emphasises delivering the utmost care aligned with evidence‐based practices and clinical guidelines. Practitioners should rely on current evidence, staying updated on research, trials and guidelines specific to wound care. Individualising treatment is crucial, considering patients' unique characteristics. Collaboration among various disciplines, including qualified wound care providers, ensures comprehensive management. Thorough assessment, considering dimensions, exudate, infection and patient symptoms, is pivotal. Patient education on wound care, participation and regular follow‐ups for plan adjustments are key, as are ethical considerations and continuous professional development. Following these guiding principles, while adhering to local and regional policies as well as national and international guidelines, helps ensure a high SOC in wound management.

Recommendation 6 Follow the “TIMERS” framework for optimal preparation of the HTHW and periwound for healing.

“TIMERS” (Tissue debridement, Infection or inflammation control/reduction, Moisture balance, Edge effect to advance epithelialisation and wound closure, Regeneration/repair of tissue to close the wound, and Social factors to be considered) is an established framework that is intended to guide clinicians in optimal assessment and preparation of the wound and periwound for healing.^7^, ^17^ “Periwound” refers to the area surrounding a wound that may be affected by wound‐related factors and/or underlying pathology.^27^

Panel members adapted the TIMERS framework to include SOC recommendations specific to CHPs and QWCPs when performing wound care. The steps for product and dressing selection within this framework are illustrated in Figure 3.

Recommendation 7 Cleanse the HTHW and periwound with a skin‐friendly cleanser.

**FIGURE 3:** General steps for product and dressing selection within the “TIMERS” framework.

Rigorous cleansing of the wound surface and periwound (including unattached non‐viable tissue) requires the active removal of skin contaminants, debris, fragments of dressings and microorganisms.^20^ The wound and periwound should be vigorously cleansed with a skin‐friendly (pH 4–6) cleanser, preferably an antiseptic solution cleanser +/− surfactant with low cytotoxicity. To ensure the area affected by the pathologies and wound‐related factors is adequately cleansed, a volume of 50–100 mL per cm of wound length is recommended.^20^, ^27^

Recommendation 8 Remove unhealthy tissue from the wound bed.

Unhealthy tissue (e.g., eschar, slough and necrotic) should be removed from the wound mechanically with gauze or a debridement pad.^30^ If gauze is painful, unhealthy tissue can be removed with debridement pads, wipes or foam. Autolytic debridement with a hydrogel, hydrocolloid, alginate, occlusive or semi‐occlusive dressing could be considered per clinician skills, patient choice and circumstances.

If available, use of a medicated/antimicrobial dressing that can impact biofilm reformation post debridement is strongly recommended. After debridement, the wound and periwound skin should be rinsed, ideally with an antiseptic solution.^18^ Antiseptic solution is preferable to saline for wound cleansing/hygiene. If sharp debridement is indicated and the required skill level or sharp instruments are not available, the patient should be referred to a QWCP. Indications for sharp debridement are listed in Table 3.

Recommendation 9 Manage infection and inflammation or refer as needed.

**TABLE 3:** Indications for when a hard‐to‐heal wound should be sharp debrided.^50^

Presence of moderate to large amount of devitalised tissue (slough, necrotic or eschar)
Debris in wound
Clinical evidence of underlying infection
Suspected biofilm
Acute cellulitis

Localised infection (biofilm) is present in the majority of HTHWs. Early intervention designed to prevent infections or treat them at the first signs is needed to switch at least a segment of these wounds back towards a healing path. All interventions to manage infection/infection risk should follow an approach based on antimicrobial stewardship principles.^20^, ^31^

Cleanse, soak and manage infection according to the level of the bioburden assessed using the wound infection continuum.^20^ An appropriate medicated/active or non‐medicated dressing with antimicrobial properties/mechanisms is recommended. Medicated wound dressings contain antimicrobial agents such as polyhexamethylene biguanide (PHMB) or medical grade honey that kill or inhibit microbial growth. Non‐medicated wound dressings have retention properties or biochemical interactions within the dressing that reduce or kill the microorganisms. Examples of non‐medicated wound dressings include dialkyl carbamoyl chloride (DACC), carboxymethycellulose (CMC), hydroconductive and super‐absorbent polymer dressings. Based on the stage of the infection continuum, for example, spreading or systemic infection, a referral may be needed for systemic antibiotic management, prescribed according to culture sensitivity and administered topically simultaneously with a medicated or non‐medicated dressing with antimicrobial properties.^32^

A standard wound culture will not identify the presence of biofilm. However, if a standard culture is taken, the Levine method is recommended, where the swab is firmly pressed down into the wound and rotated over a 1‐cm^2^ area to express fluid from the tissue.^20^

Inflammation is an indication in wounds that are at risk of infection or are infected.^32^ Although inflammation is a necessary step in the wound healing process, a commonality among hard‐to‐heal wounds is prolonged inflammation within the wounded area, even without infection.^33^ It is important to use consistent assessment tools for determining infection versus inflammation.^34^ Early recognition of the signs and symptoms of inflammation and prompt intervention are essential to enhance wound healing. Protease diagnostic testing and protease modulating dressings are recommended if appropriate.

Recommendation 10 Manage moisture in the wound and periwound to create a healthy, moist environment for healing.

Excessive exudate production or too little exudate or moisture in a wound can disrupt healing and potentially damage the periwound area. Protecting the periwound from excess moisture is key to avoiding periwound damage.^27^ The periwound is particularly susceptible to moisture‐associated skin damage (MASD) when wound drainage volume exceeds the fluid‐handling capacity of the dressing.^35^ Skin breakdown, erythema and erosion often occur in skin that has been damaged by wound exudate.^36^ Maceration may also occur when moisture is trapped against the skin for a prolonged period, which may appear as a white margin around the wound, causing the skin to soften and wrinkle.^37^

A skin barrier/liquid barrier film should be used to protect the periwound from adhesive damage, excess moisture or adhesion of non‐adhesive dressings (Figure 3). Strategies to prevent periwound damage should consist of appropriate dressing selection, sizing and correct usage, to optimise healing and limit further damage (Figure 3). CHPs should refer to a QWCP if periwound damage is complex, beyond their knowledge and skill, or persists despite good SOC.^27^ For uncontrolled periwound damage due to drainage, the patient should be referred for consideration of negative pressure wound therapy.

Recommendation 11 Apply appropriate advanced wound dressing according to wound characteristics, for example, moisture level and wound depth.

Dressing selection is an essential component of the treatment plan. The literature supports the use of moisture‐retentive dressings, such as hydrocolloids, for dry, shallow wounds. Superabsorbent, foam and alginate dressings are options for highly exudative wounds, and hydrogel dressings can benefit deeper, dry wounds that may contain nonviable tissue (Figures 3 and 4).^7^, ^38^

**FIGURE 4:** Recommended primary dressings by level of exudate (adapted from Sibbald et al.^17^).

Learning to apply and remove these dressings correctly in various clinical scenarios is essential in achieving healing. Figure 5 shows a HTHW that is returned to a positive healing trajectory with good SOC wound treatment.

**FIGURE 5:** Venous leg ulcer case study. A 63‐year‐old male presented with a recurrent venous leg ulcer on his left medial ankle (A). The periwound skin was macerated and thickened. The wound was sharp debrided and absorbent dressings were applied. Multilayer compression was applied over the dressings. After 4 months of this regimen, the wound was filled with hypergranulation tissue and healing was progressing slowly (B). The dressing was changed to an antimicrobial collagen dressing, in addition to multilayer compression (C). One week after the collagen dressings were started, the wound became considerably smaller and healthier with robust granulation tissue (D). Two weeks after the collagen dressings were started, the wound was essentially healed (E).

Although wet‐to‐dry dressings using gauze were the standard treatment for many wounds for decades, this treatment method is no longer recommended. Numerous studies have shown wet‐to‐dry gauze negatively impacts the healing environment and leads to increased risk of infection, increased dressing change frequency, greater pain at dressing changes and delayed healing. Maintaining a moist healing environment with modern dressings is considerably more effective in promoting an optimal healing environment.^30^ Gauze may still play a role in advanced wound care as a secondary dressing for low exudating wounds, or for mechanical debridement of wounds to disrupt biofilm and treat local infection when procedural pain is minimised and managed.

Recommendation 12 Arrange for compression therapy as appropriate over wounds of patients with poor venous return, including lower leg venous insufficiency ulcers.

Patients with a venous disorder, lower limb oedema, thrombosis, lymphedema or lipedema typically benefit from compression therapy in conjunction with an appropriate absorptive dressing.^39^ An ankle brachial pressure index (ABPI) test is highly recommended to determine the need for compression. If it is determined that a HTHW patient could benefit from compression, the patient should immediately be referred. If an ABPI test cannot be performed, the patient should also be referred to a QWCP for further investigation and care.

Normal ABPI range is 0.9–1.1, but ABPIs can be falsely elevated due to calcified vessels or diabetes. Patients with ABPI < 0.5 should not receive compression therapy and should be referred to a vascular surgeon for possible revascularisation.

Recommendation 13 Manage wound and periwound skin to promote epithelial advancement of the wound edges.

Adequate management of exudate, underlying pathology and bioburden are necessary to achieve epithelial advancement from the wound margins. If wound edges are rolled, cliffed or callused, appropriate debridement is recommended. If this is beyond the scope of practice, due to lack of knowledge or clinical skills, or against local policies, and particularly with respect to a periwound callus on the foot, the patient should be referred early to a wound care provider.

If tunnelling or undermining is noted, these spaces should be probed to exclude sinus or tracking, and loosely packed with selected dressing material. If this is outside the scope of practice, early referral is recommended.

Recommendation 14 Refer the repair and regeneration step of the framework to a QWCP for advanced adjunctive therapies.

If the wound has not healed or the wound size has not reduced by 40%–50% by week 4, the patient should be referred to a QWCP for advanced therapies. The aim of the repair and regeneration step is to promote wound closure by providing a matrix to support cell infiltration, stimulating cell activity using advanced adjunctive therapies including biophysical therapies, for example, negative pressure wound therapy, oxygen therapy and tissue‐based products.^40^, ^41^

Recommendation 15 Be attentive to the patient's over‐arching social situation.

Low mobility, the death of relatives and friends, an increasing lack of family cohesion and retirement can lead to feelings of social isolation and loneliness for many people with HTHWs. Pain, odour and discharge can also contribute to low self‐esteem, depression and social stigma. The link between social isolation, poor treatment adherence and low wound healing rates in patients is well documented.^42^, ^43^ Improved clinical outcomes may be achieved through CHPs who engage and empower the patient, the patient's family and others in the patient's circles of care to help care for the wound.^5^

The benefits of patient empowerment have been widely promoted in numerous programmes and publications across healthcare.^44^, ^45^, ^46^, ^47^ Getting patients to communicate their ideas, concerns and expectations about their own diagnosis and treatment exemplifies a patient‐centred approach that has been shown to provide insight into the reasons for the visit as well as to help establish the right diagnosis.^48^ Active listening by the CHP to identify patients' short‐term goals and biggest impediments to good wound care can help motivate patients and optimise treatment. Patient involvement in established social outreach groups, such as a leg club, that emphasise social interaction, participation, empathy and peer support has also been shown to positively influence wound healing and prevention.^47^ Referral for advanced pain and symptom management, and special dressings/solutions to address odour may be necessary to improve patient adherence.^5^, ^49^

Figure 6 shows a summary of recommendations for CHPs using the TIMERS framework, including optimal products to be included in wound care toolboxes for CHPs providing SOC and for QWCPs providing advanced wound care.

**FIGURE 6:** Recommended actions and toolbox items for standard of care (CHPs) and advanced wound care (QWCPs) within TIMERS framework (adapted from Sibbald et al^17^ and Atkin et al^7^).

## 4 DISCUSSION

Increases in age‐ and lifestyle‐associated conditions including diabetes, obesity and vascular disease as well as healthcare system resource limitations have contributed to a global rise in the prevalence of hard‐to‐heal wounds. Curbing the humanistic and financial burden of HTHWs increasingly involves CHPs who are often the initial contact for people with wounds. However, most literature regarding HTHWs published during the past decade is intricate and aimed at people who specialise in wound care. With current trends of nursing shortages, lack of continuity of care and fast turnover of the workforce, there is an urgent need to provide clear recommendations for CHPs who encounter wounds. The recommendations and flow charts in this document are an attempt to whittle down to the most up‐to‐date basics of SOC wound care, which if followed could considerably impact people suffering with wounds, as well as healthcare resource utilisation worldwide.

HTHWs are defined as any wound that has not healed by 40%–50% after 4 weeks of evidence‐based SOC. They occur in patients with multiple comorbidities and typically display increases in devitalised tissue, infection, exudate, maceration, wound malodour or pain, or no change in wound size. These recommendations underscore the use of person‐ and wound‐related signs to identify a HTHW and to signal the earliest possible referral to a QWCP or multidisciplinary wound care team whenever a HTHW is suspected.

When the referral process is stalled and during the period between initial wound presentation and a visit to a QWCP, these recommendations are meant to help guide CHPs in playing a critical initial role by undertaking a thorough assessment, addressing local infection and inflammation and providing an optimal wound healing environment for timely prevention and treatment of HTHWs.

Treatment recommendations for SOC include cleansing the wound and periwound with a non‐cytotoxic antiseptic or pH‐balanced surfactant solution post regional skin hygiene, followed by prompt mechanical wound debridement as appropriate. For draining wounds, the periwound should be protected with a barrier product. When increased risk of an HTHW is identified, healing is delayed or infection is suspected, a topical antimicrobial/antiseptic agent should be used. For highly draining wounds, a superabsorbent/gelling fibre dressing is recommended. Alginate or foam dressings are recommended for wounds with medium drainage, and hydrocolloid, sheet hydrogel or thin foam dressings for minimal drainage (Figure 3).

CHPs may lack appropriate products in their practice to provide good SOC wound treatment, and these recommendations suggest modest additions of basic wound care products to assemble a toolkit. According to these recommendations, a basic toolkit for wound care should include antiseptic/surfactant wound/skin cleansers, debridement products, a barrier product to protect the periwound, a selection of absorptive dressings appropriate to the level of exudate observed to ensure a moist wound environment (Figure 4), and a secondary cover dressing if needed. Armed with a toolkit and basic knowledge of SOC practices in wound care, CHPs may play an integral role in providing optimal outcomes for people with wounds.

In translating these actionable evidence‐based recommendations into practice for CHPs, several key implementation strategies should be considered. First, it is essential to facilitate easy access to the document through digital platforms and training sessions to ensure widespread dissemination among CHPs. Second, fostering a culture of continuous learning and professional development through workshops and case discussions can aid in understanding nuances of the recommendations. Third, incorporating the recommendations into electronic health record systems can serve as a digital prompt during patient encounters, helping to ensure adherence to the guidelines. Fourth, regular audits and feedback mechanisms can help monitor the application of recommendations and identify any barriers or challenges faced by CHPs. Lastly, fostering collaboration among CHPs and qualified wound care providers through multidisciplinary meetings can provide a platform for knowledge exchange, addressing queries and sharing best practices. By adopting these implementation strategies, CHPs may be empowered to identify and treat HTHWs in a manner that aligns with evidence‐based guidelines, ultimately improving patient outcomes and healthcare quality.

While these recommendations are based on best available evidence and the consensus of panel members, they do not exclude other approaches as being within a standard of practice. Adherence to any given method of wound management should be determined after taking numerous factors into account, including conditions at the relevant practice (staff levels, experience, product availability, etc.) and characteristics of the individual patient.

## CONFLICT OF INTEREST STATEMENT

Dimitri Beeckman, Emily Greenstein, Patricia Idensohn, Robert Klein, Norbert Kolbig, Kimberly LeBlanc, Catherine Milne, Terry Treadwell, Dot Weir and Wendy White are all paid consultants for 3M. Matthew Cooper is an employee of 3M.

## Data Availability

Data sharing not applicable to this article as no datasets were generated or analysed during the current study.
